# Cytotoxic and apoptogenic effect of hypericin, the bioactive component of *Hypericum perforatum* on the MCF-7 human breast cancer cell line

**DOI:** 10.1186/s12935-016-0279-4

**Published:** 2016-02-09

**Authors:** Seyed Abbas Mirmalek, Mohammad Amin Azizi, Ehsan Jangholi, Soheila Yadollah-Damavandi, Mohammad Amin Javidi, Yekta Parsa, Tina Parsa, Seyed Alireza Salimi-Tabatabaee, Hossein Ghasemzadeh kolagar, Reza Alizadeh-Navaei

**Affiliations:** 1 Department of Surgery, Islamic Azad University, Tehran Medical Sciences Branch, Tehran, Iran; 2 Students’ Research Committee, Islamic Azad University, Tehran Medical Sciences Branch, Tehran, Iran; 3 Young Researchers and Elite Club, Islamic Azad University, Tehran Medical Sciences Branch, Tehran, Iran; 4 Department of Molecular Genetics, Faculty of Biological Sciences, Tarbiat Modares University, Tehran, Iran; 5 Students Research Committee, School of Public Health, Shahroud University of Medical Sciences, Shahroud, Iran; 6 Molecular and Cell Biology Research Center, Mazandaran University of Medical Sciences, Sari, Iran; 7 Medical Research Center, Azad University, Tehran Medical Branch, Attarimoqaddam Ave, Haqani Ave, Dr. Shariati St, Tehran, P. O. BOX : 19395-1495, Iran

**Keywords:** MCF-7, Breast Cancer, Apoptosis, *Hypericum perforatum*, Hypericin, Cytotoxic

## Abstract

**Background:**

Breast cancer is the most prevalent malignancies among the women that have a high mortality. Previous studies demonstrated that hypericin, a bioactive component of *Hypericum perforatum* have a cytotoxic effect on the malignant cell lines. However, an anti-carcinogenic activity of hypericin on MCF-7 is uncertain. To investigate the cytotoxic effect of hypericin on MCF-7 cells, a human breast adenocarcinoma cell-line, that resistance to chemotherapy.

**Methods:**

The MCF-7 and fibroblast (as normal cell line) were treated with various concentrations of hypericin, and Cisplatin as a positive control for 24 and 48 h. Cytotoxicity activity was measured and confirmed by MTT assay and Trypan blue staining, respectively. In addition, Apoptosis were determined by Annexin V/Propidium Iodide assay. Immunocytochemistry (ICC) analysis for bcl2 and p53 proteins performed to further investigate different expression of these genes in different samples.

**Results:**

Both cisplatin and the hypericin exhibited a dose-dependent cytotoxic effect in the MCF-7 cell line. Although the LD50 of the hypericin was significantly lower when compared to cispaltin (5 vs. 20 μg/ml), it continued to decrease the growth rate of the MCF-7 cells when tested at higher concentration than LD50. In contrast, cisplatine, at higher concentration than LD50, completely inhibited the growth of the MCF-7 in 48 h. Regarding Annexin V/Propidium results, treatment of MCF-7 cells with LD50 concentration of cisplatin and hypericin showed 60 and 52 % apoptosis in 24 h, respectively. ICC analysis for bcl2 and p53 also confirmed our results; in treated samples for the dose of LD50 in 24 and 48 h of cisplatin and hypercin, more cells expressed p53 (guardian of cells in front of tumor formation/progression) and less expressed bcl2 (which has anti apoptotic activity) compared to untreated samples.

**Conclusions:**

Considering that hypericin showed to be cytotoxic, it seems to be a chemopreventive agent and a good candidate for antineoplastic drug development.

## Background

Breast cancer is one of the most common human malignancies, accounting for 22 % of all cancers diagnosed in women and among the most frequent causes of cancer mortality in women worldwide [1, 2]. Metastatic breast cancer is considered incurable with median survival estimates of around 2–3 years, nevertheless treatments with endocrine, cytotoxic, or targeted therapies can improve or preserve the quality of life and extend endurance. Breast cancer represents a complex and heterogeneous disease comprising distinct pathologies with specific histological features, therapeutic responses, metastatic dissemination patterns, and patient outcomes [3].

For the first time, Soule et al. [4] introduced the MCF-7 cell line, which was derived from a patient with metastatic breast cancer. Despite many studies were established MCF-7 cells as the first hormone-responsive breast cancer cell line [5]. The benefit of the MCF-7 cell line as an investigative tool led to its adoption in laboratories worldwide [5, 6]. Various evidences include the ability to undergo DNA fragmentation, differential sensitivities to estrogens and anti-estrogens, differential expression of estrogen receptors (ER), ER-mRNA, progesterone receptors and differences in tumorigenicity and proliferative rates. It has been demonstrated that the MCF-7 cell line is a novel tool for the subject area of breast cancer resistance to chemotherapy, because it seems to mirror the heterogeneity of tumor cells in vivo [7]. The human breast cancer cell line MCF-7 provides an unlimited source of homogenous self-replicating material, free of contaminating stromal cells, and can be easily cultured in simple standard media. Such a cell line is ideal to study the interaction between a chemo-preventive drug and a cancer cell. The mechanism by which a chemo-preventive drug inhibits the proliferation of a cancer cell can be better evaluated in vitro where the other physiological regulatory mechanisms, which are present in the in vivo system, are absent.

Exploring the plant chemical diversity appears to be a vital strategy for development of novel anticancer drugs characterized by alternative mode of action or lower toxicity. The intensive screening of plant-derived compounds for antineoplastic activity during the last several decades has contributed to the founding of various drug classes occupying a substantial portion of the anticancer drug market [8]. Recent evidence suggests that the members of the Guttiferae family, e.g. diverse Hypericum, Garcinia, Clusia, Cratoxylumspecies, appear to be a valuable resource of cytotoxic compounds [8–10]. *Hypericum perforatum*, known as St. John’s wort, is the most studied of Hypericum species and it is known for its pharmacological antidepressant activities, its antiviral and antibacterial properties [11, 12]. Previous phytochemical studies of *H. perforatum* revealed that the main chemical components are flavonoids, phloroglucinols and naphthodiathrones, of these, the content of flavonoids are the richest [13].

Hypericin is one of the main constitute of *H. perforatum*, which in addition to its well-known anti-depressant activity has been proven to exhibit potent cytotoxic and pro-apoptotic effects against tumor cell lines in low micro molar concentrations, and to inhibit tumor-induced angiogenesis [8, 14].

Although, extensive research has been carried out on anti-carcinogenic activity of *H. perforatum*, no single study exists which in MCF-7 cells [15–17]. Hence, this study was aimed to determine the antineoplastic activity of hypericin on human breast cell line MCF-7.

## Results

### MTT assay

To determine cytotoxicity effect of hypericin on the MCF-7 cell viability MTT assay performed. As it is shown in Fig. 1, the LD50 for 24 h for hypericin evaluated to be 5 (μg/ml); and that of cisplatin was 20 (μg/ml). Treatment of fibroblasts (as a normal cell line) with the concentrations up to 30 (μg/ml) of hypericin and/or cisplatin have not significant effect on the cells survival in 24 h (P = 0.062 and P = 0.054, respectively).

**Fig. 1:** MTT assay results for cisplatin and hypericin in 24 h on MCF-7 cell line. Treatment of MCF-7 cells with 5 (μg/ml) concentration of hypericin showed 50 % cell death (=LD50 or IC50) (**a**, *blue column*), whereas LD50 of cisplatin in this time calculated to be 20 (μg/ml) (**b**, *blue column*).*P < 0.05, **P < 0.01

LD50 for 48 h for hypericin evaluated to be 0.5 (μg/ml) (Fig. 2a); and that of cisplatin was 7.5 (μg/ml) (Fig. 2b). Interestingly cells viability increased with the increase in hypericin concentration. Treatment of fibroblasts with the concentrations up to 10 (μg/ml) of hypericin and 15 (μg/ml) of cisplatin have not significant effect on the cells survival in 48 h.

**Fig. 2:** MTT assay results for cisplatin and hypericin in 48 h on MCF-7 cell line. Treatment of MCF-7 cells with 0.5 (μg/ml) concentration of hypericin showed 50 % cell death (=LD50 or IC50) (**a**, *blue column*), whereas LD50 of cisplatin in this time calculated to be 7.5 (μg/ml) (**b**, *blue column*). * *P* < 0.05, **P < 0.01

### Flow cytometery

AnnexinV/PI flow cytometery was performed to quantify cells that underwent apoptosis after cisplatin and hypericin treatment. As it is shown in Fig. 3, treatment of MCF-7 cells with LD50 concentration of cisplatin and hypericin showed 60 and 52 % apoptosis in 24 h, respectively.

**Fig. 3:** Flowcytometery results for LD50 dose of cisplatin and hypericin in 24 h on MCF-7 cells. **a** Treatment of cells with 5 (μg/ml) concentration of hypericin showed 52 % apoptosis (*right up quadrant* shows cells in late apoptosis). **b** Treatment of cells with 20 (μg/ml) of cisplatin showed 60 % apoptosis (*cells in right up quadrant* are in late apoptosis)

### Trypan blue staining

To further investigate the effect of hypericin on MCF-7 cells death, trypan blue staining performed. After staining cells which had treated with 0.5 (μg/ml) concentration of hypericin or 7.5 (μg/ml) concentration of cisplatin for 48 h, cells became blue (Fig. 4a, b). Interestingly staining cells which had treated with hypericin in higher concentration than LD50 [>0.5 (μg/ml)] did not became blue (Fig. 4c). However, cells which had treated with cisplatin in higher concentration of LD50 [>7.5 (μg/ml)], became blue after staining.

**Fig. 4:** Staining MCF-7 cells with trypan *blue* after treatment with different doses of hypericin for 48 h. **a** and **b** MCF-7 cells which had treated with 0.5 (μg/ml) (equal to LD50 for 48 h) became *blue* after staining (**a**; ×40 and **b**; ×100). **c** MCF-7 cells which had treated with hypericin in higher concentrations than LD50 [25 (μg/ml)] did not become *blue* (**c**; ×100)

### Expression of bcl2 and p53 in different samples

To confirm that either treatment of cells with hypercin and/or cisplatin induce cell death via apoptosis and increasing p53 level and reducing bcl2 expression level, ICC for these proteins performed. As Fig. 5 demonstrates, more cells express p53 (Fig. 5), and less express bcl2 (Fig. 6) after treatment with hypercin and/or cisplatin in LD50 dose for 24 and 48 h.

**Fig. 5:** ICC staining of p53 in MCF-7 cells. ICC staining of p53 in untreated MCF-7 cells (**a**) (utilizing DAPI nuclear dye, stains cells nuclei blue [*middle columns*]). ICC results for p53 in the cells after treatment of cells with 20 (μg/ml) of cisplatin after 24 h (**b**), 7.5 (μg/ml) cisplatin after 48 h (**c**), 5 (μg/ml) of hypercin after 24 h (**d**), 0.5 (μg/ml) hypercin after 48 h (**e**). More cells are stained *green* (for p53) after treatment cisplatin and/or hypercin. (original magnification ×400; *scale bar* 50 µm)

**Fig. 6:** ICC staining for bcl2 protein in MCF-7 cells. In control samples more cells stain in *green* (**a**); compared to the samples treated with 20 (μg/ml) of cisplatin after 24 h (**b**), 7.5 (μg/ml) cisplatin after 48 h (**c**), 5 (μg/ml) of hypercin after 24 h (**d**), 0.5 (μg/ml) hypercin after 48 h (**e**). Cells nuclei become blue after counterstaining with DAPI (*middle column*). (original magnification ×400; *scale bar* 50 µm)

## Discussion

A common problem in the chemotherapy or radiotherapy of cancer is the resistance to these treatments resulting in metastasis of the malignancy. Therefore, there is a vital need to develop new anti-cancer drug [18]. Hypericin is a naturally occurring polycyclic quinone that can be extracted from the *H. perforatum* or chemically synthesized. It has been used for the photodynamic therapy of cancer and other conditions [19]. Although the mechanism of action of this compound is not known, several reports had suggested the several cellular pathways participating in the survival, necrosis, or apoptosis of the cell [19, 20]. In present study, MTT assay results for cisplatin and hypericin in 24 and 48 h on MCF-7 cell line show that LD50 of hypericin at these times was lower than cisplatin and these differences were significant. In Kim et al. study, hypericin at a concentration of 0.2 microM, exhibited 50 % growth inhibition in human myeloid leukemia U-937 cells [21]. In Hamilton et al. study, two established pituitary adenoma cell lines, AtT-20 and GH4C1, were treated with hypericin in tissue culture for defined periods following passage. Inhibition of growth was found to be dose dependent in all three cell lines in low micromolar concentrations of hypericin, as determined by viable cell counts, methylthiotetrazole assay, and [3H] thymidine uptake studies [22]. In Eriksson study, computational docking and molecular dynamics simulations are applied to investigate possible interactions between hypericin and the Ca^2+^ pump SERCA. They had shown that the transmembrane thapsigargin and butylhydroquinone binding pockets provide suitable locations for hypericin as they allow for favorable interactions with the lipid tails that enclose these. High binding energies were distinguished for hypericin in these pockets and are expected to constitute highly possible binding sites due to their accessibility from the endoplasmic reticulum membrane [23]. In Özen et al. study, hypericin was found to have cytotoxicity in HL-60 cells in time and dose dependent manner between the doses of 1 nM to 100 μM with IC50 dose of 0.5 μM. Hypericin with the dose of 0.5 μM had similar cytotoxicity pattern with the cytotoxicity curve obtained with 1/10,000 diluted extract obtained from *H. perforatum* [24]. Jendzelovsky et al. [25] show that hypericin induces the expression of two ATP-binding cassette transporters transporters: multidrug resistance-associated protein-1 and breast cancer resistance protein. Barliya et al. study, suggest that hypericin may potentially be useful in preventing growth of cancers in which hypoxia-inducible factor 1α plays pivotal roles, and in von-Hippel Lindau protein ablated cancer cells such as renal cell carcinoma through elimination of elevated hypoxia-inducible factor 1α contents in these cells, scaling down the excessive angiogenesis which characterizes these cancers [26]. Another mechanism of the hypericin, is its effect on ErbB-2. In Hwang et al. study, they used ovarian SK-OV-3 cells and investigated the effects of hypericin on the activity of the c-erbB-2 incorporation and its downstream kinases. They had shown that hypericin induce cell death with inhibition of c-erbB-2 expression and activation [27].

In the present study, apoptosis as an underlying mechanism of hypericin cytoxocity was shown by flowcytometery and ICC for bcl2 and p53 proteins. In addition, flowcytometery results for an LD50 dose of cisplatin and hypericin in 24 h on MCF-7 cells show that the rate of apoptosis in treatment of cells with 5 (μg/ml) concentration of hypericin (52 %) was lower than this rate in treatment of cells with 20 (μg/ml) of cisplatin (60 %). In Hamilton et al. study, concentrations of hypericin as low as 100 nM also induced apoptosis in these established lines, whereas treatment of normal human fibroblasts with a concentration of 10 mM failed to induce apoptosis [22]. Our ICC results confirmed these findings. In Acar et al. study, viability of cancer cells as evaluated by the XTT assay and result showed that hypericin concentration of 7.5 μg/mL led to increased apoptosis of cancer cells and finally, they demonstrated that the increase in ADAMTS1 expression may prevent metastasis or facilitate the development of an adjuvant factor with tumor-suppressive effects. Hypericin may therefore use its antitumor and apoptotic effects in MFC-7 cells via ADAMTS1 and ADAMTS3 [28]. This finding supports the idea that hypericin causes a block of the mitosis over the genome, and the apoptosis signals may originate from the genome [29]. However, Roscetti et al. [30] study, show that purified hypericin has only a weak inhibitory effect on cell growth in human erythroleukemic cell line (K562) and no effect in inducing apoptotic cell death.

## Conclusions

Results of the present study show that on MCF-7 cell line, the LD50 of hypericin was lower than cisplatin and the rate of apoptosis in treatment of cells with hypericin was lower than cisplatin. Further studies are needed to evaluate the chemo preventive potential of the hypericin when used alone or in combination with cisplatin to mitigate the toxic side effects of the latter.

## Methods

### Cell line and materials

MCF-7 cell line (NCBI No.C135, human breast cancer cell line) was purchased from Pasteur Institute of Iran (Pasteur Institute, Tehran, Iran). Hypericin (>99 %), Cisplatin and 3-[4,5-Dimethyl-2-thiazolyl]-2,5-diphenyl-2-tetrazolium bromide (MTT) assay Kit were obtained from Sigma Aldrich (USA). The cell culture plastic ware was obtained from Nunc (Denmark). High glucose Dulbecco’s Modified Eagle’s Medium (DMEM), fetal bovine serum (FBS), penicillin, streptomycin, phosphate-buffered saline (PBS) and trypsin EDTA were obtained from Gibco (USA). Annexin V-FITC apoptosis detection kit and trypan blue were s purchased from R and D systems (USA) and ACROS (New Jersey, USA), respectively. The rabbit monoclonal anti-bcl2 antibody, rabbit polyclonal anti-p53 antibody, goat anti-Rabbit IgG Fc (FITC) and 4′, 6-diamidino-2-phenylindole (DAPI) were purchased from Abcam (UK).

### Cell culture

MCF-7 cells were cultured in high glucoses DMEM supplemented with 10 % heated-inactivate FBS, containing penicillin (100 U/mL) and streptomycin (100 µg/mL) at 37 °C in a humidified atmosphere of 95 % air and 5 % CO2, and the medium was changed every other day. When the cultures were 80–90 % confluent, All cells were washed with PBS (pH = 7.4), detached with 0.25 % trypsin, centrifuged at 1200 rpm for 5 min in 37 °C and re-plated onto 96- or 24-well plates at an appropriate density according to each experimental scale. All experiments were carried out 24–48 h after the cells were plated.

Cells were seeded overnight, and then incubated with various concentrations of hypericin for 24 and 48 h. For MTT assay, cells were seeded at 8000 and 6000/well for 24 and 48 h, respectively. For each concentration and time course study, there was a control sample which remained untreated and received the equal volume of medium. All different treatment carried out in triplicate.

### MTT assay

Anti-proliferative activities of hypericin on the MCF-7 breast cancer cell line and Fibroblasts, was determined by MTT colorimetric assay [31]. Briefly, cells (8000 and 6000/well) in 200 ml DMEM containing 10 % FBS were seeded on 96-well plates and incubated overnight. These cells subsequently treated with various concentrations of hypericin, and Cisplatin as a positive control for 24 and 48 h. Afterwards, 20 μl of MTT solution (5 mg/ml in PBS) was added to each well and incubated for an additional 4 h followed by adding 200 μl of dimethyl sulfoxide. Cell viability was measured at 570 nm by an ELISA reader (Biotek ELX800 microplate reader). Lethal dose 50 (LD50) or IC50, the concentration reducing the absorbance of treated cells by 50 % with respect to untreated cells, determined by the standard curve method.

### Detection of apoptosis by flow cytometry

Apoptotic cells were determined by Annexin V/Propidium Iodide assay according to the manufacturer’s recommendation. Briefly, MCF-7 cell and Fibroblasts were cultured overnight in a 24-well plate (100,000/well) and treated with hypericin for 48 h. Floating and adherent cells were then harvested and incubated overnight at 4 °C in the dark with 750 μl of a hypotonic buffer (50 μg/ml PI in 0.1 % sodium citrate plus 0.1 % Triton X-100) before flowcytometric analysis using a FACScan flow cytometer (BD FacsCanto II, USA).

### Trypan blue staining

To confirm treatment with different dose of cisplatin or hypericin caused cell death, trypan blue staining performed. Briefly, 0.4 % trypan blue solution prepared; to eliminate background dye, after 5 min incubation of cells treated with different doses of cisplatin or hypericin (and control samples) with this solution, cells were washed with PBS. In the protocol presented here, a viable cell will have a clear cytoplasm whereas a nonviable cell will have a blue cytoplasm.

### Immunocytochemistry (ICC)

MCF-7 cells were seeded in 24-well plates. After different treatments, the cells were washed with PBS and then fixed in 4 % paraformaldehyde for 10 min at room temperature. The cells were then incubated overnight at 4 °C with rabbit monoclonal anti-bcl2 antibody or rabbit polyclonal anti-p53 antibody as primary antibodies. After this step, cells were washed with PBS three times and incubated for 1 h with FITC at 37 °C. After further washing with PBS, the cell nuclei were stained with DAPI. Staining cells without primary antibody utilized as negative. Images were captured using a laser confocal microscope (Nikon/A1 Plus, Japan).

### Statistical analysis

All results were expressed as mean ± SD The significance of difference was evaluated with ANOVA and Bonfrroni’s test. Data were analyzed by Graph Pad Prism software (version 6.01). Significant difference was set at P < 0.05.
